This article has been retracted.

# A Novel and Robust Approach to Detect Tuberculosis Using Transfer Learning

**DOI:** 10.1155/2021/1002799

**Published:** 2021-11-25

**Authors:** Omar Faruk, Eshan Ahmed, Sakil Ahmed, Anika Tabassum, Tahia Tazin, Sami Bourouis, Mohammad Monirujjaman Khan

**Affiliations:** ^1^Department of Electrical and Computer Engineering, North South University, Bashundhara, Dhaka-1229, Bangladesh; ^2^Department of Information Technology, College of Computers and Information Technology, Taif University, P.O. Box 11099, Taif 21944, Saudi Arabia

## Abstract

Deep learning has emerged as a promising technique for a variety of elements of infectious disease monitoring and detection, including *tuberculosis*. We built a deep convolutional neural network (CNN) model to assess the generalizability of the deep learning model using a publicly accessible tuberculosis dataset. This study was able to reliably detect tuberculosis (TB) from chest X-ray images by utilizing image preprocessing, data augmentation, and deep learning classification techniques. Four distinct deep CNNs (Xception, InceptionV3, InceptionResNetV2, and MobileNetV2) were trained, validated, and evaluated for the classification of *tuberculosis* and nontuberculosis cases using transfer learning from their pretrained starting weights. With an F1-score of 99 percent, InceptionResNetV2 had the highest accuracy. This research is more accurate than earlier published work. Additionally, it outperforms all other models in terms of reliability. The suggested approach, with its state-of-the-art performance, may be helpful for computer-assisted rapid TB detection.

## 1. Introduction

TB is the world's second most lethal infectious disease, trailing only human immunodeficiency virus (HIV), with an estimated 1.4 million deaths in 2019 [1]. Although it is most often associated with the lungs, it may also affect other organs such as the stomach (abdomen), glands, bones, and the neurological system. The top thirty tuberculosis-burdening countries accounted for 87% of *tuberculosis* cases in 2019 [2]. Two-thirds of the overall is made up of India, Indonesia, China, the Philippines, Pakistan, Nigeria, Bangladesh, and South Africa, with India leading the way, followed by Indonesia, China, the Philippines, Pakistan, Nigeria, Bangladesh, and South Africa. In 2019, an estimated 10 million people worldwide developed TB. There are 5.6 million men, 3.2 million women, and 1.2 million children in the country. Tuberculosis may be cured if diagnosed early and treated appropriately [3]. Almost always, *tuberculosis* can be cured with therapy. Antibiotics are often given for a six-month period [4].

Chest X-ray screening for TB in the lungs is the simplest and most frequently used technique of *tuberculosis* detection. Another alternative is to have chest radiographs examined by a physician, which is a time-consuming clinical procedure [5]. Tuberculosis is often misclassified as other illnesses with similar radiographic patterns as a result of CXR imaging, resulting in ineffective treatment and deteriorating clinical conditions [6]. In this context, a transfer learning approach based on convolutional neural networks may be critical. CXR pictures were chosen as a sample dataset in this research because they are cost-effective and time-efficient, as well as compact and readily accessible in nearly every clinic. As a consequence, fewer poor nations will profit from this study. The main motivation for this study is to diagnose *tuberculosis* without any delay. This method will aid in the fast diagnosis of *tuberculosis* via the use of CXR images. False result problems may be resolved if a model is designed with a high degree of precision. If this test were adopted, the system would be more robust and allow for the evaluation of a greater number of individuals in a shorter amount of time, significantly decreasing the spread.

### 1.1. Existing Work

Several research groups used CXR pictures to identify *tuberculosis* (TB) and normal patients using a standard machine learning method. But the objective of this article is to get a better understanding of the issue. We reviewed current papers and articles and considered strategies for improving the accuracy of our deep learning model. To compare our efforts, we utilized an existing dataset and examined their model. Using a deep learning approach, Hooda et al. classified CXR images into *tuberculosis* and non-TB groups with an accuracy of 82.09 percent. Evangelista and Guedes developed a computer-assisted technique based on intelligent pattern recognition [7]. By modifying the settings of deep-layered CNNs, it has been shown that deep machine learning techniques may be used to diagnose TB. Transfer learning was used in the context of deep learning to identify TB by utilizing pretrained models and their ensembles [8].

Pasa et al. proposed a deep network architecture with an accuracy of 86.82 percent for TB screening. Additionally, they demonstrated an interactive visualization application for patients with TB [9]. Chhikara et al. investigated whether CXR pictures might be used to detect pneumonia. They used preprocessing methods like filtering and gamma correction to evaluate the performance of pretrained models (Resnet, ImageNet, Xception, and Inception) [10]. The paper “Reliable TB Detection Using Chest X-ray with Deep Learning, Segmentation, and Visualization” was authored by Tawsifur Rahman. He used deep convolutional neural networks and the modules ResNet18, ResNet50, ResNet101, ChexNet, InceptionV3, Vgg19, DenseNet201, SqueezeNet, and MobileNet to differentiate between *tuberculosis* and normal images. In the identification of *tuberculosis* using X-ray images, the top-performing model, ChexNet, had accuracy, precision, sensitivity, F1-score, and specificity of 96.47 percent, 96.62 percent, 96.47 percent, 96.47 percent, and 96.51 percent, respectively [11].

Stefanus Kieu Tao Hwa showed deep learning for TB diagnosis using chest X-rays; according to the data, the suggested ensemble method achieved the highest accuracy of 89.77 percent, sensitivity of 90.91 percent, and specificity of 88.64 percent [12]. Priya Ebenezer et al. have extended all current TB detection proposals. They designed a new method for identifying overlapping TB items. To determine the boundaries between the single bacterium area, the overlapping bacilli zone, and the nonbacilli region, form characteristics such as eccentricity, compactness, circularity, and tortuosity were examined. A novel proposal for an overlapping bacilli area was made based on concavities in the region. Because concavities imply overlapping, the optimum separation line is determined by the concavity's deepest concavity point. This provides an additional advantage. When the separation is overlapped, the overall count of *tuberculosis* bacilli is much more precise [13]. Vishnu Makkapati et al. were the first to diagnose TB using the form characteristics of *Mycobacterium tuberculosis* bacteria. They proposed a method based on hue color components for segmenting bacilli through adaptive hue range selection. The existence of a beaded structure inside the bacilli, as well as the thread length and breadth parameters, indicates the validity or invalidity of the bacilli [14]. Sadaphal et al. developed a method in 2008 that incorporated (1) Bayesian segmentation, which relied on prior knowledge of ZN stain colors to estimate the likelihood of a pixel having a “TB item,” and (2) shape/size analysis [15].

In the majority of studies, researchers claimed around 90% accuracy. However, the major contribution of this research is that several pretrained models were utilized. InceptionV3 was 96 percent accurate and 97.57 percent validated, MobileNetV2 was 98 percent accurate and 97.93 percent validated, and InceptionResNetV2 was 99 percent accurate and 99.36 percent validated. This study presents a novel method for detecting tuberculosis-infected individuals using deep learning.

CNN (convolutional neural networking) is a technique that is well suited for this kind of issue. This method will aid in the rapid detection of *tuberculosis* from chest X-ray pictures.

The remaining portion of the article is organized as follows: Section 2 addressed the approach and methodology. Sections 3 and 4 addressed the analysis of the results and the conclusion, respectively.

## 2. Method and Materials

Open-source Kaggle provided the dataset used in this study. Patients with *tuberculosis* and those without the disease were represented in the dataset. For feature extraction, a CNN is used. A flatten layer, two dense layers, and a ReLU activation function are all included in the model. It also includes four Conv2D layers and three MaxPooling2D layers. SoftMax, the last and most thick layer, serves as an activation layer. Transfer learning is also utilized in this study to compare the accuracy of the created model with the accuracy of the pretrained model. With a few changes in the final layers, MobileNetV2, InceptionResNetV2, Xception, and InceptionV3 were utilized for pretrained models. Layers such as average pooling, flatten, dense, and dropout are used to create bespoke end results. When it comes to extracting visual details, the CNN model works effectively. The model learns and distinguishes between images by extracting characteristics from the input images.  Figure 1 shows the workflow diagram of the TB and normal image detection.

*Python* is the perfect programming language for data analysis. Because of *Python*'s extensive library access, deep learning problems are very successful in the *Python* programming language. On a personal GPU, Anaconda Navigator and Jupyter Notebook were used for dataset preparation, as well as Google Colab for handling large datasets and online model training.

### 2.1. Dataset

This system's dataset is made up of 3500 TB and 3500 normal images. For this study, the Tuberculosis (TB) Chest X-ray Database has been used [16]. The visualization of this dataset is shown in Figures 2 and 3.

Figure 2 depicts a healthy chest X-ray, whereas Figure 3 depicts a disease chest X-ray caused by *tuberculosis*. The pictures in the collection have varying starting heights and widths. Those provided pictures have a predetermined form thanks to the model. The Tuberculosis (TB) Chest X-ray Database is a balanced medical dataset. The total number of *tuberculosis* and nontuberculosis cases is equal (3500 each).  Figure 4 displays the total number of TB and non-TB records in this dataset.

### 2.2. Block Diagram

A dataset with two subsections is provided as input in the block design shown in Figure 5. This system underwent some preprocessing before fitting the model, such as importing pictures of a certain size, dividing the dataset, and using data augmentation methods. Better accuracy was achieved after fitting and fine-tuning the model. It was possible to see how loss and accuracy evolve over time by plotting a confusion matrix and a model of loss and accuracy. As a final step, the classification result section shows how well the model did in distinguishing between pictures of TB and those not associated with the disease.

The entire system is shown in the block diagram in the simplest possible manner. In this research, the decision-making component of the system plays a very important role. An enormous quantity of data is used to train the model, which then uses that data to make a conclusion.

### 2.3. Preprocessing

The preprocessing phase occurs before the training and testing of the data. Picture dimensions are redimensioned, images are transformed to an array, input is preprocessed using MobileNetV2, and hot labels are finally encoded throughout the four preparation stages. Because of the effectiveness of the training model, picture scaling is an important preprocessing step in computer vision. The smaller the image, the smoother it runs. In this research, an image was resized to 256 by 256 pixels. Following that, all of the images in the dataset will be processed into an array. For calling, the image is converted into a loop function array. The image is then used in conjunction with MobileNetV2 to preproceed input. The last step is hot coding on labels, since many computer learning algorithms cannot operate directly on data labelling. This method, as well as all input and output variables, must be numerical. The tagged data are transformed into a numerical label in order to be interpreted and analyzed. Following the preprocessing step, the data are divided into three batches: 70 percent training data, 20 percent validation data, and the remaining testing data. Each load contains both normal and TB images.

Several increments were used to add variety to the original images. Because lung X-rays are generally symmetrical with a few minor characteristics, increases such as vertical images were used. However, the main goal was for TB and associated symptoms to occur in either lung and be detectable in both of our models. To provide more variety, these improved images have been gently rotated and illuminated or dimmed.

### 2.4. Convolutional Neural Network and Transfer Learning

In artificial intelligence, CNNs (convolutional neural networks) are often employed for image categorization [17]. Before the input is sent through a neural network, it handles data convolution, maximum pooling, and flattening. It works because the various weights are set up using various inputs. Once the data have passed through the hidden layers, weights are computed and assessed. Following input from the cost function, the network goes through a back propagation phase [18]. During this procedure, the input layer weight is readjusted once again, and the process is repeated until it finds an optimal position for weight adjustment there. Epochs show how many times the cycle has repeated itself. It takes a long time to train a model using neural networks, which is a major disadvantage. To get around this, we will utilize transfer learning, another hot subject in computer vision research [19]. To learn from a dataset, we use transfer learning, which makes use of a pretrained model. It saves us a lot of time in training and takes care of a lot of different important things at the same time. As time passes, we will be able to fine-tune our networks for improved accuracy and simplicity.

Transfer learning is to preserve knowledge from one area and apply it to another. Training takes a long time since model parameters are all initialized using a random Gaussian distribution and a convergence of at least 30 epochs with a lot of dimensions of 50 pictures is generated. The problem stems from the fact that big, well-noted pictures may be difficult to obtain in the medical profession. Due to a paucity of medical data, it is sometimes difficult to correctly predict models. One of the most difficult problems for medical researchers is the shortage of medical data or datasets. Data are an important factor in deep learning methods. Data processing and labelling are both time-consuming and costly. The advantage of transfer learning is that it does not require vast datasets. Computations are becoming easier and less costly. Transfer learning is a technique in which the knowledge from a pretrained model that was trained on a large dataset is transferred to a new model that has to be trained, incorporating fresh data that is comparatively less than needed. For a specific job, this method started CNN training with a tiny dataset, which included a large-scale dataset that had previously been trained in the pretrained models.

### 2.5. Overview of the Proposed Model

Four CNN-based pretrained models were used in this research to classify chest X-ray pictures. Xception, InceptionV3, MobileNetV2, and InceptionResNetV2 are the models used. There are two types of chest X-ray pictures: one is unaffected by *tuberculosis*, whereas the other is. This study also utilized a transfer learning technique that can perform well with sparse data by utilizing ImageNet data and is efficient in terms of training time. The symmetric system architecture of the transfer learning method is shown in Figure 6.

InceptionResNetV2 was developed by merging two of the most well-known deep convolutional neural networks, Inception [20] and ResNet [21], and using batch normalization rather than summation for the traditional layers. The popular transfer learning model, InceptionResNetV2, was trained on data from the ImageNet database from various sources and classifications, and it is definitely making waves. When include top = “False”, it simply indicates that the fully connected layer will not be included, even if the input shape is specified. 224 × 224 × 3. When training = “False”, the weights in a particular layer are not changed during training. The dropout layer, which aids in overfitting prevention, randomly sets input units to 0 at a rate frequency at each step during training time. Dropout (0.5) represents a dropout effect of 50 percent. Flattening is the process of converting data into a one-dimensional array for use in the next layer. The output of the convolutional layers is flattened to generate a single large feature vector. It is also linked to the final classification model, forming what is known as a fully connected layer. Batch normalization is a method for improving the speed and stability of artificial neural networks by recentering and rescaling the inputs of the layers. When building the pretrained models, Table 1 indicates that the batch size is 32, the maximum epoch is 25, and a loss function of “binary cross-entropy” is used.

The sigmoid function is an activation function that assists a neuron in making choices. These routines produce either a 0 or a 1. It employs probability to generate a binary output [22]. The outcome is determined by determining who has the highest probability value. This function outperforms the threshold function and is more useful for categorization. This activation function is often applied to the last dense block. The equation for the sigmoid function is

(1) $$\begin{array}{c} X=\frac{1}{1+e^{-Y}}. \end{array}$$

ReLU is an activation function that operates on the concept of rectification. This function's output stays at 0 from the start until a specified point. After crossing or reaching a certain value, the output changes and continues to rise as the input changes [23]. Because it is only activated when there is a significant or significant input inside the neurons, this function works extremely well.

### 2.6. Evaluation Criteria

Following the completion of the training phase, all models were evaluated on the test dataset. The performance of these systems was evaluated using the accuracy, precision, recall, F1-score, and AUC range. This study's performance measures are all mentioned below. True positives (TP) are *tuberculosis* images that were correctly identified as such; true negatives (TN) are normal images that were correctly identified as such; false positives (FP) are normal images that were incorrectly identified as *tuberculosis* images; and false negatives (FN) are normal *tuberculosis* images.

Accuracy simply indicates how close our expected result is to the actual result [24]. It is represented as a percentage. It is determined by adding true positive and true negative and dividing the overall number of potential outcomes by the number of possible outcomes:

(2) $$\begin{array}{c} \text{Accuracy}=\frac{\text{TP}+\text{FN}}{\text{TP}+\text{TF}+\text{FP}+\text{FN}}. \end{array}$$

Precision is a measure of how close predicted outcomes are to each other [25]. True positive is obtained by dividing true positive by the sum of true and false positives:

(3) $$\begin{array}{c} \text{Precision}=\frac{\text{TP}}{\text{TP}+\text{FP}}. \end{array}$$

Recall is determined by dividing the total number of true positives by the total number of true positives and false negatives:

(4) $$\begin{array}{c} \text{Recall}=\frac{\text{TP}}{\text{TP}+\text{FN}}. \end{array}$$

The F1-score combines a classifier's accuracy and recall into a single measure by calculating their harmonic mean. It is most commonly used to compare the results of two different classifiers. Assume classifier A has greater recall and classifier B has greater precision. In this case, the F1-scores of both classifiers may be used to determine which performs better. The F1-score of a classification model is computed as follows:

(5) $$\begin{array}{c} F1=\frac{2\left(\text{Precision }x\text{ Recall}\right)}{\text{Precision}+\text{Recall}}. \end{array}$$

It evaluates the correctness of the model dataset. Although accuracy is difficult to grasp, the F1-score idea becomes more useful in situations of uneven class distribution. It is used by many machine learning models. It is utilized when false negatives and false positives are more important in the dataset than genuine positives and true negatives. When the data are wrongly categorized, it produces better results.

The confusion matrix displays the total number of right and erroneous outcomes. It is possible to see all true-positive, false-positive, true-negative, and false-negative numbers [26].The greater the frequency of genuine positive and true-negative outcomes, the greater the accuracy.

## 3. Result and Analysis

In classifying normal images and TB, we experimented with a variety of models and methods in order to assess their utility and efficacy. Four pretrained CNN models were employed to classify chest X-ray pictures. The models that are relevant include MobileNetV2, Xception, InceptionResNetV2, and Inception V3. There are two kinds of chest X-ray pictures. The first is TB, whereas the second is normal. This study also used ImageNet data to use a transfer learning method that is successful in terms of training times when there is insufficient data.

Several network designs, including Xception, InceptionV3, InceptionResNetV2, and MobileNetV2, are tested before deciding on a network architecture. A bespoke 19-layer ConvNet is also tried, but it performs badly. The InceptionResNetV2 performed the best of all networks, and the findings based on that design are included.  Table 2 shows the accuracy and loss history of four tried models.

According to Table 2, the InceptionResNetV2 model achieves a validation or testing accuracy of 99.36 percent, with a validation loss of 2.37 percent. Normal images have 99 percent accuracy, 98 percent recall, and 99 percent F1-scores, whereas TB images have 98 percent precision, 99 percent recall, and 99 percent F1-scores.

Figures 7 and 8 indicate that, at epoch 1, the training accuracy was pretty low in the first few epochs. The starting training accuracy is 57.20 percent, the training loss is 69.01 percent, the validation accuracy is 74.79 percent, and the loss is also huge (905.03 percent), indicating that the model learns very slowly at first. The training accuracy improves as the number of epochs increases and the loss function begins to decrease. The model evaluates the results at the end of 25 epochs; InceptionResNetV2 has a 99.12 percent train accuracy and a 99.643 percent validation accuracy, with a train loss of 3.40 percent and a validation loss of 1.71 percent.

In identifying normal and tuberculosis (TB) images, Figure 9 illustrates true-positive, true-negative, false-positive, and false-negative scenarios.

According to the results, the InceptionResNetV2 model correctly identifies images as “normal” 98 percent of the time and incorrectly labels normal photos as “TB” 2 percent of the time. Additionally, the confusion matrix shows that the algorithm accurately classifies 99 percent of TB photographs as “TB,” while predicting 1 percent of photographs as “normal.”

Additionally, this research included genuine testing, which provided input to the model through chest X-ray images. When the model is complete, a file with the hdf5 extension is created containing the produced model. Four hdf5 files representing four different models were created for this study. Following that, a new notebook file is created with the ipynb test extension. Four models were included in this test file, and then, individual chest X-ray images were provided as input. Figures 10 and 11 show the prediction results in real time.

The result shown in Figure 10 is normal. The input image was normal, and the model correctly predicted it.  Figure 11 shows a *tuberculosis* chest X-ray image as an input. The model then returned a valid result, indicating that the input picture was of a TB chest X-ray. In Table 3, classification results have been compared with the above reference papers.

In this article, using MobileNet, we achieved 97.93 percent accuracy, but in [11], the authors achieved 94.33 percent accuracy by using the same algorithm. But the difference between their work and our work is that we fine-tuned the model to increase its accuracy, whereas they used the general MobileNet algorithm in their work. Using InceptionV3, they achieved higher accuracy than our model, but overall in this article, InceptionResnetV2 achieved the highest accuracy of 99.36 percent, which is greater than any previous work reported before.

## 4. Conclusion

A framework for deep learning analysis may be very beneficial for individuals who do not get regular screening or checkups in countries with insufficient healthcare facilities. Deep learning in clinical imaging is particularly apparent in early analyses that may recommend preventive therapy. Due to a shortage of radiologists in resource-limited areas, technology-assisted *tuberculosis* diagnosis is required to help reduce the time and effort spent on *tuberculosis* detection. Medical analysis powered by deep learning is still not as remarkable as experts would want. This study suggests that we may approach that the level of accuracy by integrating many recent breakthroughs in deep learning and applying them to suitable situations. In this research, we utilized the pretrained model InceptionResNetV2 to develop an automated *tuberculosis* detection method. With a validation accuracy of 99.36 percent, the InceptionResNetV2 model has finally reached the new state of the art in identifying *tuberculosis* illness. Given the following, an automated TB diagnosis system would be very helpful in poor countries where trained pulmonologists are in limited supply. These approaches would improve access to health care by reducing both the patient's and the pulmonologist's time and screening expenses. This advancement will have a profound effect on the medical profession. Tuberculosis patients may be readily identified with this method. Diagnostics will benefit from this kind of approach in the future. Numerous deep learning methods may be used to improve the parameters and generate a trustworthy model that benefits mankind. Additionally, we may experiment with a number of image processing techniques in the future to aid the model in learning the picture pattern more accurately and provide improved performance.

## Figures and Tables

**Figure 1:** Workflow diagram of the TB or normal image detection.

**Figure 2:** Non-TB X-ray images.

**Figure 3:** Tuberculosis X-ray images.

**Figure 4:** Total number of TB and non-TB records.

**Figure 5:** Block diagram of the proposed system.

**Figure 6:** System architecture with InceptionResNetV2.

**Figure 7:** Training and validation accuracy.

**Figure 8:** Training and validation loss.

**Figure 9:** Confusion matrix.

**Figure 10:** Normal prediction.

**Figure 11:** TB prediction.

**Table 1:** Parameters used for compiling various models.

Parameters	Value
Batch size	32
Shuffling	Each epoch
Optimizer	Adam
Learning rate	1*e*^−3^
Decay	1*e*^−3^/epoch
Loss	Binary_crossentropy
Epoch	25
Execution environment	GPU

**Table 2:** Comparison of pretrained models.

Model	Train accuracy	Val accuracy	Train loss	Val loss	Images	Precision	Recall	F1-score
Xception	0.9596	0.9543	0.1155	0.1213	Normal	1.00	0.90	0.95
					TB	0.91	1.00	0.95
InceptionV3	0.9800	0.9757	0.1160	0.1243	Normal	0.95	0.97	0.96
					TB	0.97	0.95	0.96
MobileNetV2	0.9930	0.9793	0.0220	0.0548	Normal	0.96	1.00	0.98
					TB	1.00	0.96	0.98
InceptionResNetV2	0.9912	0.9936	0.0340	0.0237	Normal	0.99	0.98	0.99
					TB	0.98	0.99	0.99

**Table 3:** Model comparison with other research.

This paper (model name)	Accuracy (%)	References paper (model name)	Accuracy (%)
MobileNet	97.93	Ref [11] MobileNet	94.33
	(Validation or testing)		
InceptionV3	98.00	Ref [12] InceptionV3	83.57
		Ref [11] InceptionV3	98.54
Xception	95.96	Ref model VGG16	87.71
InceptionResNetV2	99.36	Ref [12] Model ChexNet	96.47
	(Validation or testing)	Ref [12] Model DenseNet201	98.6
MobileNet	97.93	Ref [27] GoogleNet	89.6

## Data Availability

The data utilized to support these research findings are accessible online at:https://www.kaggle.com/tawsifurrahman/tuberculosis-tb-chest-xray-dataset.
